The article "Complex Survival System Modeling for Risk Assessment of Infant Mortality Using a Parametric Approach" was published in 2022. Journal: Comput Math Methods Med.

# Complex Survival System Modeling for Risk Assessment of Infant Mortality Using a Parametric Approach

**DOI:** 10.1155/2022/7745628

**Published:** 2022-04-19

**Authors:** Hang Chen, Maryam Sadiq, Zishen Song

**Affiliations:** ^1^Department of Electronics and Information, Xi'an Jiaotong University, Shaanxi 710049, China; ^2^Department of Statistics, University of Azad Jammu and Kashmir, Muzaffarabad, Pakistan

## Abstract

Pakistan is still one of the five countries contributing to half of the child deaths worldwide and holds a low ratio of infant survival. A high rate of poverty, low level of education, limited health facilities, rural-urban inequalities, and political uncertainty are the main reasons for this condition. Survival models that evaluate the performance of models over simulated and real data set may serve as an effective technique to determine accurate complex systems. The present study proposed an efficient extension of the recent parametric technique for risk assessment of infant mortality to address complex survival systems in the presence of extreme observations. This extended method integrated four distributions with the basic algorithm using a real data set of infant survival without extreme observations. The proposed models are compared with the standard partial least squares-Cox regression (PLS-CoxR), and higher efficiency of these proposed algorithms is observed for handling complex survival time systems for risk assessment. The algorithm is also used to analyze simulated data set for further verification of results. The optimal model revealed that the mother's age, type of residence, wealth index, permission to go to a medical facility, distance to a health facility, and awareness about tuberculosis significantly affected the survival time of infants. The flexibility and continuity of extended parametric methods support the implementation of public health surveillance data effectively for data-oriented evaluation. The findings may support projecting targeted interventions, producing awareness, and implementing policies planned to reduce infant mortality.

## 1. Introduction

Strong statistical survival techniques are the demand of the era for authentic and reliable results for deeply examining complex survival and mortality patterns. Nonparametric survival techniques including the Kaplan-Meier product-limit method [1], the Gehan's generalized Wilcoxon test [2], and the log-rank test [3] were extensively used in older times. The Cox's regression model remained the most popular and widely used semiparametric survival technique if the proportional hazards assumption is fulfilled [4]. In recent times, flexible parametric models (FPM) are considered as a better alternative to nonparametric and semiparametric methods as they produce estimates with higher efficiency and lower standard errors [5]. In addition, these models consider full likelihood to draw more precise inferences and easily interpretable results. So far, the FPM has been employed various probability distributions to estimate survival functions. The exponential probability distribution supports as the baseline to handle survival time. The Weibull, Gompertz, generalized gamma, and generalized F-distribution are commonly practiced too. The FPM is also able to efficiently investigate the relationship of covariates with survival response [5]. The partial least squares-Cox regression (PLS-CoxR) integrates PLS with the Cox model to address survival time response with collinear covariates [6] since the Cox regression is restricted with inflexible estimates of the cumulative hazard and survival functions as being incomplete. Hence, the PLS-CoxR model is restricted in the long-term estimation with unsmooth functions.

The flexible parametric models (FPMs) are recommended to compute hazard and cumulative hazard functions for covariates to extrapolate the survival model. The FPM can estimate continuous survival and hazard functions instead of a step representation due to its flexibility [7].

Despite considerable improvement towards increasing infant survival, nearly six million child deaths are recorded every year, before attaining their fifth birthday [8]. By the end of 2015, a minor proportion of developing countries have met the fourth target of Millennium Development Goal (MDG) which is intended to increase the child survival rate by two-thirds [9]. The recently described Sustainable Development Goals (SDG) seek to forward the objectives originated by the MDG. The third SDG is to reduce the under-five mortality rate (U5MR) to 25 deaths per 1000 live births by 2030 [10]. Previous literature evidenced that five countries including China, Congo, Nigeria, India, and Pakistan possess nearly half of under-five mortality in the world [11]. Pakistan has the sixth largest population in the world with 188 million people [12]. In 2018, Pakistan's infant mortality rate (IMR) was 61 deaths per 1000 live births. Due to political instability, civil conflicts, poverty, lower educational level, unavailability of health facilities, and disparities regarding the area in Pakistan, 70% MDG targets were not achieved [13]. Understanding the factors affecting infant mortality is significantly informative to health professionals, practitioners, and health policymakers for the improvement of population health status through effective interventions.

Within this line, the partial least squares flexible parametric model (PLS-FPM) is developed to analyze the complex survival systems in the presence of extreme observations for risk and hazard assessment [14]. The present study extended the PLS-FPM to collinear predictors having moderate trend observations using four alternative probability distributions.

The results exposed the flexible dynamics of the extended method to obtain smooth survival and hazards estimates in the presence of multicollinearity. This model can be implemented in the field of genetics, biology, engineering, medicine, social sciences, or behavioral sciences for system reliability and risk assessment. The formal statements of the problem are the following:

- Selection of optimum model by execution of four distribution integrated with the PLS-FPM oversimulated and real data set having collinear predictors and moderate observation
- Identification of significant risk factors of infant mortality in Pakistani

## 2. Methodology

The PLS-CoxR model is considered as the benchmark method in the present study, and the PLS-FP model with four different distributions is the proposed technique.

### 2.1. The Cox Regression Model

The Cox model has the form

(1) $$\begin{array}{c} \lambda \left(t\right)=\lambda_{o}\left(t\right)\exp\left(\beta_{1}X_{1}+\beta_{2}X_{2}+\cdots +\beta_{p}X_{p}\right)=\lambda_{o}\left(t\right)\exp\left[\beta^{\prime }X\right], \end{array}$$

where *λ*_*o*_(*t*) represents the baseline hazard function, *β* is the vector of regression estimates, and *X* denotes a (*n*∗*p*) matrix of predictors.

### 2.2. The Partial Least Squares-Cox Regression Model

The PLS-CoxR model is employed as the reference method in the present study. Suppose the survival time is represented by *t* and *x*_*j*_ = *x*_1*j*_, *x*_2*j*_, ⋯, *x*_*nj*_ be the vector of *p* correlated covariates with *n* samples. The model estimates *k* components for *p* correlated predictors and assumes the hazard estimate as

(2) $$\begin{array}{c} \lambda \left(t\right)=\lambda_{o}\left(t\right)\exp\left(\beta_{1}S_{1}+\beta_{2}S_{2}+\cdots +\beta_{p}S_{k}\right)=\lambda_{o}\left(t\right)\exp\left[\beta^{\prime }S\right], \end{array}$$

where *S* represents a (*n*∗*k*) matrix of components.

### 2.3. Flexible Parametric Survival Model (FPSM)

Let *T* represent a nonnegative continuous survival response and let *X* is the vector of predictors *x*_1_, ⋯, *x*_*p*_ over a sample of size *n*. The survival function is the probability of being alive at time *t* and is represented by *S*(*t*) = *Pr*(*T* > *t*) for a vector of covariates at time *t* with the cumulative distribution function *F*(*t*) = *Pr*(*T* ≤ *t*). Then the cumulative hazard or risk function is

(3) $$\begin{array}{c} \Lambda \left(t\right)=\int_{0}^{t}\lambda \left(x\right)dx. \end{array}$$

Any distribution ranges over *t* ∈ [0, ∞], and it may serve as survival distribution. The survival distributions included in this study as FPSM are as follows:

#### 2.3.1. The Gompertz Distribution

A survival response *T* following a Gompertz distribution with parameters (*b* > 0, *η* > 0) exhibits the survival function

(4) $$\begin{array}{c} S\left(t\right)=\exp\left(-\frac{b}{\eta }\left(e^{\eta t}-1\right)\right), \end{array}$$

and the cumulative hazard function as

(5) $$\begin{array}{c} \Lambda \left(t\right)=\frac{b}{\eta }\left(e^{\eta t}-1\right). \end{array}$$

The Gompertz distribution is also an extreme value distribution with increasing hazard function.

#### 2.3.2. The Generalized Gamma Distribution

The generalized gamma distribution with parameters (*β*, *σ*, *κ*) has survival function as

(6) $$\begin{array}{c} S\left(t\right)=1-\Gamma \kappa^{-2}\left(e^{-\beta }t{}^{\kappa /\sigma };\kappa^{-2}\right]. \end{array}$$

The hazard function of the generalized gamma function is increasing, decreasing, bathtub, and arc-shaped [15].

#### 2.3.3. The Generalized F-Distribution

The density function of generalized F-distribution with 2*ν*_1_ and 2*ν*_1_ is

(7) $$\begin{array}{c} f\left(t\right)={\left(\nu_{1}e^{t}/\nu_{2}\right)}^{\nu_{1}}{\left(1+\nu_{1}e^{t}/\nu_{2}\right)}^{-\left(\nu_{1}+\nu_{2}\right)}\beta {\left(\nu_{1},\nu_{2}\right)}^{-1}, \end{array}$$

where *β*(*ν*_1_, *ν*_2_) is the beta function and then the survival function is

(8) $$\begin{array}{c} S\left(t\right)=\int_{0}^{\nu_{2}{\left(\nu_{2}+\nu_{1}e^{t}\right)}^{-1}}\chi^{\nu_{2}-1}{\left(1-\chi \right)}^{\nu_{1}-1}\beta {\left(\nu_{2},\nu_{1}\right)}^{-1}dx, \end{array}$$

where *χ* denotes the chi-square distribution. This distribution is useful for testing different parametric forms as it includes other distributions as limiting or special cases.

#### 2.3.4. The Exponential Distribution

The survival time *T* has an exponential distribution with rate parameter *λ* having density function

(9) $$\begin{array}{c} f\left(t\right)=\lambda \exp\left(-\lambda t\right), \end{array}$$

then the survival function is

(10) $$\begin{array}{c} S\left(t\right)=\exp\left(-\lambda t\right), \end{array}$$

and the cumulative hazard function is

(11) $$\begin{array}{c} \Lambda \left(t\right)=\lambda t. \end{array}$$

Several other probability distributions can be employed in FPM. The interpretation for regression coefficients of FPM is the same as for semiparametric models. The FPM provides a more stabilized cumulative hazard function than the semiparametric model. For instance, the Weibull models produce the hazard function as a continuous straight trend. The PLSR model integrated with FPM addressing generalized gamma (GG), generalized F (GF), exponential, and Gompertz distribution is included in the present study for improved model performance for multicollinear covariates.

### 2.4. The Partial Least Squares Flexible Parametric (FP) Model

The proposed model assumes the occurrence of an event *e* at time *t* in the presence of censoring, and let *X* be the matrix of *p* correlated predictors *x*_1_, ⋯, *x*_*p*_ for a sample of size *n*. The method computes the FP model for *S* components (as *S* ≤ *p*) computed from PLSR for survival response and *X* as a matrix of predictors. The PLS-FP model assumes that some *A* is equal to the number of components to be predicted (where *A* ≤ *p*), then for *a* = 1, 2, ⋯, *A*, the algorithm runs:

1. Loading weights are computed by

(12) $$\begin{array}{c} w_{a}=X\prime_{a-1}t_{a-1}. \end{array}$$

Loading weights are normalized to have length equal to 1 by

(13) $$\begin{array}{c} w_{a}⟵\frac{X_{a-1}^{\prime }t_{a-1}}{\left\|X_{a-1}^{\prime }t_{a-1}\right\|}. \end{array}$$

(2) Score vector *s*_*a*_ is computed by

(14) $$\begin{array}{c} s_{a}=X_{a-1}w_{a}. \end{array}$$

The risk function for FPSM is computed as

(15) $$\begin{array}{c} \Lambda \left(t\right)=\int_{0}^{t}\lambda \left(s\right)ds. \end{array}$$

(3) If *a* < *A* return to 1

The PLS-FP model is a two-stage procedure. At the first stage, the PLS-FP regression model computes components of PLS regression with time as response outcome and correlated covariates as predictors. Then, it executes the FP model with survival time as response and components of PLSR as explanatory factors at the later stage. This method produces efficient estimates with increased accuracy for collinear predictors. Hence, it is recommended to use in the case of collinear data as it is a conjugate of PLS and FP models. The PLSR model is also coupled with a filter-based factor selection method, namely, “loading weights” to identify the significant factors [16, 17].

### 2.5. Simulated Survival Data Generated from Gompertz Distributions

The R-package namely “simsurv” is used for the generation of simulated survival data [18] with moderate observation and collinear predictors. The data follows Gompertz distribution with 0.1 and 0.1 scale and shape parameters, respectively. The correlation among predictors is established as (0.9, 0.8, 0.7, 0.6, 0.5, 0.4, 0.3, 0.2, 0.1, 0) for 100 samples with 30 predictors.

### 2.6. Infant Survival Times Data

This study used secondary data, obtained from the Demographic and Health Surveys (DHS), gathered during 2012-2013 from Pakistan. Hence, no ethical concerns are required to conduct this study [19]. The present analysis used data set of infants aged 1-12 months in Pakistan. Due to missing and incomplete information, infants dead within one month of birth are excluded from the analysis. A total of 697 infants belonging to Pakistan and 83 predictor variables are included.

## 3. Results

The PLS-FPM parameterized with generalized gamma, generalized F, exponential, and Gompertz distribution are modeled on simulated data generated from Gompertz distribution to observe the variation in efficiency for multicollinear data. The left panel of Figure 1 showed the efficiency of models established by AIC and indicated that coupled with PLSR, the FPM models showed the higher efficiency over simulated data having known correlation structure. Similar results based on BIC, as shown in Figure 1(b), are observed. The simulation analysis demonstrated that the proposed models are efficient and reliable in terms of performance for the corresponding distributions. The analysis over simulation recommended the practical application of proposed models to examine survival response along with correlated covariates in a more flexible manner.

Before analyzing the real data set, multicollinearity among covariates is verified to justify the application of PLS. For this purpose, correlations structure for infant survival data is examined. The biplot for infant survival data presented in Figure 2 clearly portrayed the correlation between covariates showing close points of occurrence.

Real data set of infant survival with 12 months of censoring is considered in this analysis. Discarding outliers, 83 covariates measured over 577 observations (infants) were included in the final sample to compare survival models. The data set is randomly split into testing (30%) and training data (70%) for reliable results. After verification of multicollinearity among covariates, the PLS-FPM parameterized over Gompertz, generalized gamma, generalized F, and exponential distribution are analyzed. The PLS-Cox model for survival time is considered as the reference method.  Figure 3 showed the efficiency of models measured by AIC and BIC which demonstrated the higher performance of modified models compared to the PLS-Cox over infant survival data. The proposed models based on the parametric approach performed better due to their additional flexibility. Flexible parametric models integrated with PLSR parameterized with generalized gamma (GG), generalized F (GF), exponential, and Gompertz distribution showed increased accuracy compared to the Cox model integrated with PLS.

The Gompertz distribution is modeled into the innovation-imitation paradigm, and its hazard function works as a convex function. These properties develop their flexibility to use as flexible parametric distribution in survival models. Hence, it increased the performance of the model incorporated with PLS compared to the semiparametric model, due to its flexible nature. Based on AIC and BIC, it is concluded that the PLS-FPM parameterized over generalized F (GF) is the best-fitted model and hence further executed for influential factor selection. PLS-FP model based on generalized F-distribution with location parameter *μ* is found to be the most efficient model over infant survival times data. In this model, covariates on the corresponding parameter represent the accelerated failure time (AFT) model which speeds up or slows down the passage of time. A detailed illustration of PLS-FP model parameterization is presented in Table 1 to describe the corresponding location, scale, shape, and rate parameter of the associated distribution.

Figure 4 showed the cumulative hazards regression estimates for the reference method and the PLS-FPM integrated with generalized gamma (GG), generalized F (GF), exponential, and Gompertz distribution for infant mortality data. The proposed PLS-FPM delivered smooth regression coefficients of the hazard functions extrapolated to a time of 12 months showing consistent estimates. The reference model showed unsmooth hazard trends with odd fluctuations for certain time intervals shown in Figure 4.

For modeling the survival time data, the PLS-FPM parameterized over generalized F (GF) is applied, and a well-known factor selection method of PLS, namely, loading weights, is used to estimate the regression coefficients of significant factors. The estimates of important predictors associated with infant mortality are presented in Table 2.

After analysis, 28 influential factors out of 80 which significantly affect infant survival in Pakistan are observed. A negative relationship of mother's age, region, selection for domestic violence, main roof material, relationship to household head, wealth index, availability of mosquito bed net, awareness about tuberculosis (TB), decision power to visit family, preceding birth interval, duration of breastfeeding, blood relation with husband, and total pregnancy outcomes are found for infant survival. Furthermore, positive association of province, mother's education, toilet facility, availability of television, sex of household head, shared toilet, number of total children, number of dead son and daughters, use of contraception, availability of permission, money, transport, and attendant for medical facility and distance to a medical facility was observed.

## 4. Discussion

Estimating the hazard and survival functions that flexibly explain complex systems remained a hard and computationally challenging task. Hence, the candidate models are usually limited in studies to allow for evaluations and comparisons. However, nonparametric and semiparametric survival methods can peculate model structures as unsmooth estimates are evaluated. The present study extended the PLS-FPM [14] to correlated predictors having moderate trend observations using four alternative probability distributions. The PLS-FPM extends previous survival approaches that either perform semiparametric analyses or use nonparametric methods, while analysis of all previous methods was limited due to their inflexible nature. To administrate all four shaped hazard functions, distribution fitting is implemented over defined simulated survival data set.

Most previous literature used the Cox regression model for infant survival analysis [20]. Very few recent studies used FPM to examine infant survival analysis [21]. The PLS-FPM is compared with the reference method for both simulated and a real data set for collinear covariates. A previous study proposed the PLS-FPM integrated with Gamma, Weibull, log-logistic, and log-normal distributions for data with extreme observations to examine four real data sets of breast cancer survival time and identify the significantly associated gene signatures for each data set. The study found that the PLS-FPM has higher performance than the traditional PLS-Cox model [14]. Consistent with the previous study, the present study found the higher efficiency of the PLS-FPM compared to the PLS-Cox regression method for data sets with moderate observations. The PLS-FPM coupled with Gompertz distribution is found to be the optimum model to estimate hazard functions using AIC for simulated survival data following Gompertz distribution. The efficiency of the algorithms flexibly increases the model accuracy to a greater extent even considering correlated predictors. This accuracy suggested that hazard, as well as survival functions, can be accurately computed by smooth trends for the survival response. A recent study proposed the partial least squares spline modeling approach by integrating PLS with restricted cubic spline model and compared it with the PLS-Cox model [22]. The study estimated the risk factors of infant mortality in Pakistan by using the PLS-spline model based on the odds scale with one knot. This study also examine the important factors of infant mortality by executing the optimal model, namely, the PLS-FPM parameterized over generalized F (GF), and identified the influential factors which are also determined by various previous studies. Consistent with the recent literature, the present study evidenced that mother's age, region, selection for domestic violence, relationship to household head, wealth index, awareness about tuberculosis (TB), decision power to visit family, preceding birth interval, and blood relation with husband [22] are significantly associated with infant mortality. Some other previous literature also supported the association of main roof material [23, 24], availability of mosquito bed net [25], duration of breastfeeding [26], and total pregnancy outcomes [27] with infant survival similar to the present study.

Various previous studies also observed the positive association of province [28], mother's educational level [29], type of toilet facility [30], availability of television [31], sex of household head [32], shared toilet [33], number of total children [34], number of died son and daughters [35], use of contraception [36], and availability of permission, money, transport, distance and attendant for medical facility [37, 38] with infant survival which is consistent with the current study. Last but not least, the PLS-FPM not only can extrapolate survival response besides the availability of follow-up information but also sponsors variant hazard shapes. The PLS-FPM is suggested as a helpful parametric addition for the estimation and prediction of survival response. This model is recommended to use in reliability theory for risk assessment.

## Figures and Tables

**Figure 1:** The comparison of the PLS-Cox model with the PLS-FPM parameterized over generalized gamma (GG), generalized F (GF), exponential, and Gompertz distribution for simulating survival response generated from Gompertz distribution based on AIC and BIC.

**Figure 2:** A biplot visualizing the correlations between the covariates on the first two principal components for infant survival data set.

**Figure 3:** The comparison of reference model with the PLS-FPM parameterized over generalized gamma (GG), generalized F (GF), exponential, and Gompertz distribution on the basis of AIC and BIC for infant survival are presented.

**Figure 4:** The cumulative hazard estimates of the PLS-Cox and the PLS-FPM parameterized over generalized gamma (GG), generalized F (GF), exponential, and Gompertz distribution for infant survival data.

**Table 1:** A description of corresponding parameter of each distribution used in the PLS-FPM for infant survival data set is presented.

	Parameter			
Model	Location	Scale	Shape	Rate
*FPM*_*pls*_*gomp*	—	—	0.231	-7.20
*FPM*_*pls*_*gg*	4.32	-0.32	0.56	—
*FPM*_*pls*_*gf*	4.37	-1.44	-0.11, 2.96	—
*FPM*_*pls*_*g*	—	—	0.77	-3.56

**Table 2:** The coefficient estimates of influential factors for infant survival obtained by the PLS-FPM coupled with GF-distribution.

Factor	Coefficient
Mother's age	-0.2599634
Province	0.1152137
Type of place of residence	-0.2259600
Selected for domestic violence module	-0.1314814
Mother's educational level	0.1150733
Type of toilet facility	0.1306607
Household has: television	0.1123271
Main roof material	-0.1824950
Relationship to household head	-0.1462302
Sex of household head	0.1263040
Toilet facilities shared with other households	0.1128781
Wealth index	-0.2221866
Total children ever born	0.1440127
Sons died	0.1444297
Daughters died	0.1380171
Used contraceptive methods	0.1255910
Have mosquito bed net for sleeping	-0.1472814
Getting medical help for self: getting permission to go	0.2765390
Getting medical help for self: getting money needed for treatment	0.1091858
Getting medical help for self: distance to health facility	0.2711795
Getting medical help for self: having to take transport	0.1405939
Getting medical help for self: not wanting to go alone	0.1932727
Heard of tuberculosis or TB	-0.2165038
Person who usually decides on visits to family or relatives	-0.1273039
Preceding birth interval (in months)	-0.1647803
Duration of breastfeeding	-0.1697750
Blood relation with husband	-0.1285042
Total pregnancy outcomes	-0.1926369

## Data Availability

Data is freely available at https://dhsprogram.com/.
